# Design and development of human resource management computer system for enterprise employees

This article has been retracted.

**DOI:** 10.1371/journal.pone.0261594

**Published:** 2021-12-17

**Authors:** Tianqi Wang, Ning Li, Houran Li

**Affiliations:** 1 School of Logistics, Linyi University, Linyi, Shandong, China; 2 Economic Management College, Pingdingshan University, Pingdingshan, Henan, China; 3 School of Marxism, Linyi University, Linyi, Shandong, China; Ministry of Natural Resources North Sea Bureau, CHINA

## Abstract

Client-Server (C/S) application is always used in the existing Human Resource Management System (HRMS) as the system architecture, which has the problems of complex maintenance and poor compatibility; and cannot use professional database and development system, making the system development difficult and the data security low. To solve the above problems, the overall demand is analyzed, as well as feasibility and key technologies of the enterprise HRMS system. Then a HRMS is designed and developed, based on the user’s key functional requirements and related technologies, which is reasonable and easy to maintain. The system is supported by Browser-Server (B/S) structure, with the current popular Java 2 Platform Enterprise Edition (J2EE) multi-level structure as the overall architecture. The mature Microsoft SQL Server 2008 introduced by Microsoft is used as the database platform. Combined with Model View Controller (MVC) design pattern, this system can be used by users without geographical restrictions and system maintenance. In this system, performance logic and business logic are separated, which makes it convenient for the development and maintenance of the system. The system mainly includes six modules: personnel management, organizational management, recruitment management, training management, salary management and system management, which integrates enterprise information and realizes the functions of easy access and easy query of information database. Its interface is simple, easy to understand, and easy to operate, with low investment, low cost, high safety, good performance and easy maintenance, which help to improve the work efficiency and modern management level of enterprises. In the end, the operation performance of the system is tested. The results show that the throughput of the main functional modules in the system is greater than 100 times/s when dealing with the business, and the success rate of event processing is greater than 99%. The average response time of the business end is less than 0.4 s, and the average response time of the terminal side is less than 0.5 s, which all meet the standards. System CPU occupancy rate can be basically controlled below 30%, and memory usage rate is below 30%. In summary, the system designed here has the basic functions but also to ensure good performance, suitable for enterprise personnel management, organizational management, recruitment management, training management and salary management. The design and development of this system aims to provide technical support for the service quality of enterprise human resource management business, to improve the overall efficiency, promote the pace of enterprise strategic development, and enhance the market competitiveness of enterprises.

## Introduction

With the development of science and technology, computer and network technology are becoming more and more developed. Computer plays an irreplaceable role in various fields of human society. Enterprise competition is no longer limited to the market, but also gradually closer to the network. Enterprise management has gradually entered the track of informalization [1]. Talent is a key factor for enterprises to achieve their strategic goals and an important issue related to their survival and development [2]. The reform of enterprise management system has never stopped, talent competition has become a new challenge to human resources [3]. In order to stand out in the fierce competition, enterprises must have a high level of talent management. The traditional human resource management is in a manual mode, which has the problems of low work efficiency, insufficient data delayed update, scattered resources, and poor sharing. Manual human resource management has been unable to meet the needs of both supply and demand of human resources with diversified and multiple organizational structures [4]. Therefore, the design and development of Human Resource Management System (HRMS) is imperative, in order to make enterprise human resource management more scientific and efficient, improve the level of enterprise informatization and market competitiveness, and retain and absorb talents better [5].

Rafidah and Dewi (2020) pointed out that the focus of human resource management should be made on recruiting and cultivating the best talents to ensure so that the quality of company personnel would be in the best state. Based on the theory of human resource management [6], Gao (2020) discussed the concrete practice of human resource management system in manufacturing enterprises. The results showed that a good human resource management system could improve the company’s production capacity and income, effectively improve the enthusiasm of employees, and be conducive to improving the ability of enterprises to withstand risks [7]. Zheng (2020) expounded the innovation of human resource management mechanism in colleges and universities based on computer aided technology. The analysis results show that the human resource management system in colleges and universities must be innovated in order to promote the development of higher education [8]. Abdullah et al. (2020) proposed and implemented an enterprise human resource management system model, using cloud technology to solve human resource problems in this field. The system is developed by using CodeIgniter and other technologies as a software framework, and started and deployed on the Amazon Web Service (AWS) elastic computing cloud [9]. To sum up, the reasonable design and development of HRMS is helpful to mobilize the enthusiasm of the staff, and improve the production capacity and income of enterprises, which plays an important role in human resource management.

Existing HRMS uses the C/S application as the system architecture. Although C/S architecture has the advantages of fast response and high security, its maintenance is complex and poor compatibility, which cannot meet the practical needs. Besides, the system data management and extraction does not use professional database. So, its security cannot be guaranteed. Based on the above background, a reasonable and easy to maintain human resource management computer system is designed and developed. This system uses Browser-Server (B/S) structure as the support. The system takes the current popular J2EE multi-level structure as the overall architecture, uses Microsoft SQL Server 2008 as the system database platform, combined with MVC design pattern, which facilitates the development and maintenance of the system. The innovation of lies in substituting the traditional C/S architecture with the B/S architecture, making users work without geographical restrictions and client maintenance; J2EE development system is adopted with high compatibility with B/S architecture to simplify the system development process; the high-security and high-efficiency Microsoft SQL Server 2008 database combined with MVC design pattern is applied to the system to achieve the safety management of data, convenient extraction, and the separation of performance logic and business logic. The paper elaborates and analyzes the system demand, feasibility, key technology, system design and development, and function realization effect, aiming to provide technical support for the service quality of enterprise human resource management business. The research also helps to improve the overall work efficiency, to promote the strategic development of enterprises, and to enhance the market competitiveness of enterprises.

## Materials and methods

### Analysis of computer system of human resource management

#### 1. System requirements analyses

(1) Users requirements analyses. The main functions of the system are as follows: 1. The system can provide staff information, contracts information and file information for the personnel department. 2. Organizational Commissioner users can use this system to invoke organizational structure, information query, modification and other functions of existing posts and vacant posts, and timely adjust in accordance with business and organizational changes. 3. The system can provide comprehensive tracking and recording functions for content promotion, resume reception, interview appointment, employment approval, notification and other links for enterprise recruitment. 4. The system can provide staff salary accounting and management, salary data recording, staff personal tax and social security expenses accounting, welfare payment schedule recording and open staff query permissions for remuneration commissioners. 5. The system can provide training commissioners with comprehensive tracking of training course deployment, lecturer and venue appointment, planning time, information announcement and other processes, as well as training effect, feedback and opinion record. 6. This system can make human resources management more efficient through collaboration between different modules [10].

(2) Performance requirements analyses. 1. The interface should be easy to operate. Window style and color design of interface are reasonable and easy for users to operate the system, through which the business and software are easy to handle. 2. Safety. It is necessary to ensure that the data in the system is not tampered or stolen by illegal intrusion, and to avoid the damage of data information due to the failure of the system itself. 3. The software is easy to upgrade and maintain. The corresponding functions of the system can be modified following the development of enterprises and policy changes. It should have certain adaptability. 4. Stability. It is necessary to ensure the rapid response and data transmission of the system when used by a large number of users. And it is also necessary to ensure the security and stability of the system [11].

#### 2. System feasibility analyses

(1) Technical feasibility analyses. The system is supported by B/S structure, which can realize the office of users without geographical restrictions and maintenance of the system. With the widely used J2EE multi-level structure as the overall architecture, JavaEE technology can provide a variety of open source, free and mature plug-ins, which can be compatible with Linux or Windows systems, and easy to operate. Microsoft SQL Server 2008, developed by Microsoft and highly integrated with the Internet, is used as the system database platform to provide guarantee for data security of enterprise. MVC design pattern is selected to realize the separation of performance logic and business logic, which facilitates the development and maintenance of the system.

(2) Economic feasibility analyses. The software and related hardware of this system are all designed by the common computer system software and hardware in the market, which can be used just by one computer, one printer and one related maintenance system software. The maintenance of the system does not require professionals, and can be completed by using the system software, which saves a lot of costs in operation and maintenance.

(3) Operation feasibility analyses. The system can smoothly access the required operation of the target server by inputting relevant passwords on any computer that can access the Internet. It does not need to operate and download special software on the specified computer, which is convenient for operators to use.

### Key technology analyses of the system

#### 1. Design of system’s architecture

C/S mode is server-centered, which can make full use of the hardware advantages of server and client, allocate tasks reasonably and reduce the communication time of the system. The client can obtain the required network resources by accessing the server, and the information uploaded by the client can be stored on the server. Fig 1 demonstrates the C/S system’s architecture.

**Fig 1:** C/S system’s architecture.

B/S refers to an improvement of C/S, also known as a triple-layer C/S architecture. The B/S structure only needs a browser to solve the problem that special software must be used in the traditional way to operate, which greatly saves the cost and simplifies the development, maintenance and use of the system. It is a new software system developing technology. This model unifies the client and focuses the core parts of the system functions on the server. As long as a browser is installed on the client and a database is installed on the web server, data interaction can be realized [12]. Fig 2 shows the structure of B/S system.

**Fig 2:** Structure of B/S system.

By using B/S structure, system and software can have the server to complete the installation, modification and maintenance functions. The biggest advantage of B/S structure is that whenever and wherever you want a computer that can connect to the Internet, you can achieve the purpose of accessing the client without installing any special software. Both structures have advantages and backwards, as shown in Figs 3 and 4 [13].

**Fig 3:** Comparison between advantages of B/S architecture with C/S architecture.

**Fig 4:** Comparison between disadvantages of B/S architecture with C/S architecture.

Although C/S architecture has the advantages of fast response and high security, its maintenance is complex and poor compatibility, which cannot meet the practical needs. Therefore, after a comprehensive comparative analysis, B/S is selected as the architecture of HRMS.

#### 2. MVC design pattern

MVC design pattern is a mature architecture pattern in the current Web development. It divides Web applications into three levels: Model (model layer), View (view layer) and Controller (control layer). When the interface and data need to be improved, it will not be necessary to rewrite the business logic and greatly optimizes the code [14]. The model layer is usually responsible for the database access operation, which is used to process data logic in the application system. The view layer is mainly used for data display, which is established based on the data model. The controller is mainly used to read the data of the view layer, and send the data to the model layer to process the man-machine interaction design in the application system. MVC plays a significant role in system development, which can be understood as a company-oriented model. Fig 5 shows the framework.

**Fig 5:** Structure of MVC.

#### 3. J2EE technology

J2EE technology is based on Java2 platform, providing technical support for the simplification of enterprise system and software development, management and deployment of complex problem architecture [15]. It is introduced to overcome the shortcomings of the traditional C/S model, conform to the development trend of the B/S structure, and enable the development and design based on Java technology to obtain a more ideal and standardized enterprise-level platform. The architecture of J2EE is mainly composed of client layer, web layer, business logic layer and enterprise information system layer. J2EE is based on a multi-tier distributed application model. The application logic is divided into components according to functions. Components are software units with independent functions. They are assembled into J2EE applications through related classes and files, and interact with other components [16]. Fig 6 shows J2EE structure and component technology.

**Fig 6:** J2EE structure and component technology.

J2EE platform can run normally in the conventional Web. In the stage of system development and design, J2EE architecture and MVC mode are selected, and the three-tier architecture based on B / S is used as a support to ensure good stability and advanced technology. At the same time, the system is strongly easy to use [17].

#### 4. UML modeling technology

Unified Modeling Language (UML) is a language for visual modeling of software-intensive systems, which uses image symbols as the modeling language to describe all aspects of the system. UML modeling charts are usually composed of a number of squares and boxes, connectors and texts, which seem to be simple but play a very important role [18]. UML diagrams are divided into use case view, design time view, process view, implementation view, and topology view, as Fig 7.

**Fig 7:** Basic classification of UML diagrams.

Among them, the use case diagram is the first step in the whole process from the analysis of system requirements to the final realization. It describes the system functions from the perspective of users, and points out that the performers of each function and the functions that the system needs to complete for the performers [19]. The use case diagram contains three basic components: participants, use cases, and relationships.

1. Participants. Persons dealing with the system are represented by human icons.
2. Use cases. A complete function of the system is represented by an ellipse.
3. Relationship. Relationships are defined between use cases, such as generalization, extension, and inclusion.

#### 5. Microsoft SQL Server 2008 database

Microsoft SQL Server is a comprehensive database platform launched by Microsoft, which has the advantages of convenient use, strong scalability and practicability, and high software integration [20]. Microsoft SQL Server2008 is the most powerful and comprehensive version of Microsoft SQL Server. This platform has the following characteristics:

1. Dependability. Applications that enable enterprises to run the most critical tasks have higher security, reliability and scalability.
2. High efficiency. It can reduce the time and cost for enterprises to develop and manage data infrastructure.
3. Intelligence. As a comprehensive and flexible development platform, it can provide relevant data information when users need them [21].

The core components of Microsoft SQL Server 2008 include the following four categories:

1. Database engine. It is mainly used for data storage, management, access control and transaction processing operations.
2. Analysis service. It provides support for online analysis and data mining in existing databases.
3. Report service. It gives report presentation of generating classified summary information based on existing data and enables users to access reports and use data.
4. Integration services. Data, processing results and data processing reports in core components are integrated to achieve data integration. Fig 8 shows architecture of Microsoft SQL Server 2008.

**Fig 8:** Architecture of Microsoft SQL Server 2008.

### Design and development of system

#### 1. Logic structure of the system

The logical structure of the system is the ideological classification of the whole system, the system is divided into a number of logical units, respectively, to achieve their functions, the development of the system makes an important decision. With the help of the logic structure of the system, we can judge the logic elements and their connections that the system composition should contain. The focus can be attracted on the function, which covers the visible/implied two kinds of functional modules in the system. The system is layered, and the orderly operation of various business processes is realized through the collaboration of each layer [22]. A typical HRMS computer system should be divided into three levels from the functional level: basic data layer, business processing layer and decision support layer.

1. Basic data layer. It mainly includes the static data which usually changes little. The data are divided into employee personal attribute data and enterprise data. This layer can save and transform information of different modules, and map different types of relational model to object model through database, so that the system has powerful and effective information access function.
2. Business processing layer. System functions that include specific business processes of human resource management are used to implement different business logic processing, complete analysis processing of user request, and use data layer to persist information processing. This layer is the main data source for enterprises to master the status of human resources, improve the human resources management and provide decision support.
3. Decision support layer. It is presented directly to the end user, which can accept operation and request of the user, also can display the final result. Users can quickly obtain the required information through the statistical analysis data of this layer, which not only improves the efficiency of human resource management, but also helps senior managers to grasp the human resources situation. Fig 9 shows the logic of the system.

**Fig 9:** Logic of the system.

#### 2. Function module design of the system

Based on the results of system requirements analysis, the paper constructs a perfect and effective HRMS. According to the key functional requirements of user, the system is divided into the following six functional modules:

1. Human resource management. It is aimed at the comprehensive management of employees, covering the management of various information from their entering the duty to their exiting the duty. So that these kinds of information are structured, standardized and systematized, to realize the query, modification, deletion, addition, statistics and other operations of various information of employees, which can improve the efficiency of human resource management, and reduce human, material and time costs [23].
2. Organizational management. It is mainly an important part of the management of enterprise system architecture. It is necessary to carry out comprehensive management of existing positions, as well as the management of vacant positions in enterprises, so as to generate a report of vacant positions and provide a reference for the recruitment plan. At the same time, according to the structure of the organization and job types of enterprises, the staff should be assigned into the corresponding vacancy departments and positions, so as to promote the comprehensive management of organizations, staff, departments and positions, and contribute to the coordination and deployment of subsequent planning [24].
3. Recruitment management. Recruitment is the most basic part of human resource management. The management of enterprises can be directly seen from the quality of recruitment management. Enterprise recruitment management is mainly to track, record and manage the recruitment process of new employees, and form a close relationship with management of organization. According to the information provided by the vacancy report, managers formulate recruitment plans, publish recruitment information, and complete the tracking and recording of resume reception, interview and written examination invitations, and entry approval [25].
4. Training management. It is a key part that cannot be ignored in the human resource management system. It covers the tracking records of many sections such as training needs analysis, plan formulation, curriculum arrangement, organization and implementation, training feedback and opinions. It realizes the organic connection with human resource information, scientific training management, and provides scientific basis for the allocation of human resources and the promotion of employees in enterprises [26].
5. Salary management. It covers the accounting and management of employee salary, the record of salary data, the accounting of employee personal tax and social security expenses, the record of welfare payment progress and the opening of employee inquiry rights. It helps enterprises to establish a sound salary management system, simplify the salary accounting process, improve work efficiency and mobilize the enthusiasm of employees. Fig 10 signifies the use case diagrams for 5 major management modules.
6. System management. It contains adding and management of user information. It controls and manages the permissions of different users to use the system. Different permissions correspond to the access interface of different information units, and provide information resources to different users.

**Fig 10:** Use case diagrams for 5 major management modules (a. use case diagram of personnel management; b. use case diagram of organization management; c. use case diagram of recruitment management; d. use case diagram of training management; e. use case diagram of remuneration management).

### Methods of system test

#### (1) Success rate of event handling

The success rate (*SR*) of the human resource management system designed is calculated as Eq (1)).

$$SR=\frac{P_{s}}{P_{s}+P_{f}}$$ (1)

In Eq (1):

*P*_*s*_ represents the total times of successful system events handling;

*P*_*f*_ represents the total times of failed system events handling.

#### (2) Transactions Per Second (TPS)

Transactions Per Second (*TPS*) refers to the times of requests that the system processes of users per unit time. It is one of the most important means in network maintenance and fault detection. The *TPS* index mainly reflects the ability of the server to withstand pressure and its load capacity. Eq (2) shows the calculation of *TPS*:

TPS=CN/ART (2)

In Eq (2):

*CN* represents the Concurrent Number;

*ART* represents the Average Responding Time.

#### (3) Occupancy Rate of CPU

Central Processing Unit (CPU) occupancy rate refers to the proportion of CPU resources occupied by the program running in the machine, which represents the situation that the machine runs the program at a certain time point. Eq (3) shows calculation of the CPU Occupancy Rate (*OR*) of the system during operation.

$$OR=\frac{T_{c}}{T_{f}}=\frac{CPI\times IC}{T_{f}}$$ (3)

In Eq (3):

*IC* represents Instructions of Computer;

*T*_*f*_ represents Clock Frequency;

*T*_*c*_ represents Clock circle.

*CPI* represents Circles of Per Instruction of computer. Eq (4) shows the calculation of *CPI*.

$$CPI=\sum_{i=1}^{n}\left(CPI_{i}\times P_{i}\right)=\sum_{i=1}^{n}\left(CPI_{i}\times \frac{IC_{i}}{IC}\right)$$ (4)

In Eq (4):

*P*_*i*_ represents the periodicity of using the instructions *i*;

*CPI*_*i*_ represents Circles of Per Instruction *i*;

*n* represents the number of the classes of instructions;

*IC*_*i*_ represents the number of instructions for class *i* instructions.

## Results

### Realization effect of main functions of the system

#### 1. Login module

The login module is used to verify the legitimacy of the user. The system can be entered after verification, so as to prevent illegal users from entering the HRMS. The user enters the system by entering the user name and password created by the administrator. Fig 11 shows the login page.

**Fig 11:** Realization effect of login page of the system.

#### 2. Human resource management

Personnel management is used to input, query, add, modify and delete all the information of enterprise staff from entering the duty to exiting the duty. Fig 12 shows the interface of human resource management.

**Fig 12:** Realization effect of human resource management.

Fig 12 manifests that after entering the personnel management page of the system, the administrator needs to enter the employee’s certificate, the employee ’s work number in the company, the date of birth, gender, the postal code of the location, the bank account number of the payroll card, the employee’s educational background and the information of the graduating school, family address, contact mode, the current department in the company and the position of the employee for later query and deletion.

#### 3. Organization management

Organizational management is a comprehensive management of enterprise architecture and job information, including comprehensive information of various departments, existing positions and vacant positions, so that enterprises can adjust and deploy relevant departments and positions in a timely manner in the development process. Fig 13 shows the interface of the organizational management.

**Fig 13:** Realization effect of the interface of the organizational management.

#### 4. Recruitment management

Recruitment management is the most basic part of HRMS, which is mainly used to track and record the recruitment process of new employees, including recruitment content promotion, resume reception, appointment interview and entry approval. Fig 14 shows the interface of the recruitment management.

**Fig 14:** The interface of the recruitment management.

#### 5. Training management

Training management is an important part of HRMS, which is mainly used to track the whole process of enterprise training, including training plan, training implementation, training feedback and opinions. Fig 15 shows the interface of training management.

**Fig 15:** The interface of training management.

#### 6. Salary management

Salary management is mainly used for the accounting, recording and managing of wages and insurance of employees. It includes compensation accounting and management, wage data records, employee tax and social security cost accounting, welfare payment schedule records and open query permissions of employees. Fig 16 shows the interface of the salary management.

**Fig 16:** The interface of the salary management.

### Performance of the system

In the system performance test, 100 users operate the system at the same time. Fig 17 show the results of performance test.

**Fig 17:** Results of performance test (a. Test results of throughput of system in business processing host and success rate of event processed; b. test results of average response time in business processing end and average response time in terminal side; c. test results of CPU occupancy and memory occupancy in system operation).

Fig 17A manifests that, the system’s personnel management, organizational management, recruitment management, training management and compensation management of the five major functional modules in the processing of business host throughput are 101.36 times/s, 102.28 times/s, 100.67 times/s, 100.29 times/s, and 101.59 times/s; more than 100 times/s. Besides, the success rates of event processing are 99.5%, 99.7%, 99.7%, 99.6% and 99.8%, respectively; more than 99%, the success rate is high. Fig 17B shows that the average response time of the terminal side of the 5 functional modules is 0.34s, 0.4s, 0.38s, 0.35s and 0.29s, respectively, which is maintained below 0.5s. The average response time of business-side processing is 0.24s, 0.31s, 0.29s, 0.21s and 0.26s, respectively, which is less than 0.4s and meets the standard. Fig 17C indicates that the CPU occupancy rates of the five functional modules in the system are 25%, 19%, 21%, 29% and 17%, respectively, which are less than 30%. The memory occupancy rates are 20%, 22%, 11%, 27% and 15%, respectively, and are all below 30%. In summary, the system designed here has excellent throughput, event processing ability, and response speed. When dealing with business, its CPU and memory occupancy rates are low, which is suitable for application in enterprises to improve the overall efficiency and management quality.

## Conclusions

Talent management is the key section for enterprises to stand out in the fierce market competition. It is very important to have a high level of human resource management. At the beginning, analyzation is made on the overall needs, feasibility, and key technologies of enterprise HRMS system. Then based on the user’s key functional requirements and related technologies, a reasonable and easy to maintain HRMS is designed and developed. The system mainly includes six modules: personnel management, organizational management, recruitment management, training management, salary management and system management, which integrates enterprise information and realizes the functions of easy access and easy query of information database. Interface simple, easy to understand, easy to operate; low investment, low cost, high safety, good performance and easy maintenance, these factors within the system can make it improve the work efficiency and modern management level of enterprises. In the end, the operation performance of the system is tested. The results show that the throughput of the main function modules in the system is greater than 100 times/s when dealing with the business, and the success rate of event processing is greater than 99%. The average response time of the business end is less than 0.4s, and the average response time of the terminal side is less than 0.5s, which all meet the standards. System CPU occupancy rate can be basically controlled below 30%, memory usage rate is below 30%. In summary, the system designed here has the basic functions but also to ensure good performance, suitable for enterprise personnel management, organizational management, recruitment management, training management and salary management. The deficiency is that the system is still in the design and developing stage, and it is not used in the actual enterprise work. Whether it is suitable for most enterprises remains to be further verified. In the future, this system should be promoted and tested in different types of enterprises. In this process, the function and performance of the system should be continuously improved according to the needs of different enterprises and the problems found. The design and development of this system aims to provide technical support for the service quality of enterprise human resource management business, improve the overall efficiency, promote the pace of enterprise strategic development, and enhance the market competitiveness of enterprises.

## Supporting information

S1 File (ZIP)
